RETRACTED

# Exploring the Medication Pattern of Chinese Medicine for Peptic Ulcer Based on Data Mining

**DOI:** 10.1155/2021/9072172

**Published:** 2021-11-11

**Authors:** Guigui Li, Youlei Guo

**Affiliations:** ^1^Second Department of Spleen and Stomach Diseases, Gansu Provincial Hospital of Traditional Chinese Medicine, Lanzhou City 730050, Gansu, China; ^2^Department of Anorectal Diseases, Gansu Provincial Hospital of Traditional Chinese Medicine, Lanzhou City 730050, China

## Abstract

During the last decades, Chinese medicine has been widely used for curing various diseases in the healthcare domain. Based on the databases of medicine wisdom and modern application of prescriptions, we have explored the medication pattern of ancient and modern prescriptions for the treatment of peptic ulcer in various patients. In this paper, we have proposed a neural network model which is based on the time series decomposition and is able to mine and predict the medication pattern of peptic ulcer treatment in Chinese medicine. For this purpose, cumulative distance level method, Mann–Kendall trend analysis, Hurst exponent, and characteristic point methods are used for the trend analysis. Likewise in the proposed model, the wavelet analysis method is used for the periodicity analysis and Mann–Kendall mutation test method along with Pettitt methods is used for mutability analysis. In addition, autocorrelation and unit root methods are utilized to test the random terms. The Chinese herbal formulas (where the main diseases are peptic ulcer, peptic ulcer, cerebral leakage, and cerebral abscess) are collected from the databases of medicine wisdom and modern application of prescriptions. Furthermore, methods of frequency analysis, association rule analysis, and factor analysis are used to evaluate the grouping pattern of prescriptions for peptic ulcer treatment. The error in the proposed scheme between the predicted and the measured values of 87 prescriptions, which involve five Chinese medicines for peptic ulcer and 160 Chinese medicines, obtained from the neural network was 16.79%.

## 1. Introduction

Peptic ulcer is a chronic disorder of the gastrointestinal system which is caused by the erosion of the gastrointestinal mucosa by gastric acid and pepsin. It is divided into gastric and duodenal ulcers with respect to the site of predilection. The clinical manifestations are chronic, periodic, and rhythmic epigastric pain with acid reflux and belching [1]. Its pathogenesis is complex and variable and it is often associated with serious complications, which are thought to be related to HP infection, gastric acid and pepsin erosion, nonsteroidal anti-inflammatory drugs, mental stimulation, and genetics. There is no name for peptic ulcer in Chinese medicine, but according to its symptoms, location, and complications, it is generally classified as “gastric pain,” “acid reflux,” “gastric gangrene,” and “noisy” in Chinese medicine. The symptoms of peptic ulcer are generally classified as “gastric pain,” “acid reflux,” “gastric distention,” and “noisy” in Chinese medicine, but “gastric pain” is more common.

RETRACTED

The clinical research on diseases of the spleen and stomach system has been carried out for many years. In practice, we have continuously inherited, developed, and innovated and have our own unique insights into the Chinese medical evidence-based treatment of peptic ulcer, focusing on the combination of disease and evidence and flexible treatment. The development of the disease is similar to that of surgical canker sores, and it is highly likely that the treatment is based on the theory of canker sores such as clearing heat and dampness, likewise, eliminating canker sores and creating muscles, supporting the root of the disease as the treatment method, and integrating the method of eliminating, supporting, and replenishing in the diagnosis and treatment of ulcer disease. In order to achieve the effect of spleen ascending and stomach descending, Qi and blood harmonization, remembering that “one point of stomach qi is kept, one point of vitality,” and not forgetting to cultivate the middle qi at the same time of treatment, we get good results every time.

Therefore, Chinese medicine treatment is said to have a long history and rich literature and many clinical experiences and medication rules need to be urgently excavated and summarized. MedicineWise is a leading medicine database in China, which contains a large number of ancient medical texts and their prescriptions [2, 3]. The Prescription Modern Application Database of the National Population and Health Science Data Sharing Platform contains nearly 10,000 Chinese medicine prescriptions derived from the Chinese Pharmacopoeia, Chinese Prescriptions, and various literature and journals [4]. Based on the above two databases, this study collected ancient and modern prescriptions for peptic ulcer treatment, analyzed their medication patterns using various data mining methods, and provided references for Chinese medicine treatment of peptic ulcer.

Data mining or prediction has been conducted on the medication used in the treatment of peptic ulcer in Chinese medicine, without establishing a close connection between data mining and prediction. Data mining provides information support for data prediction and results are verified. Accuracy of data mining are complementary to each other. Since the medication for peptic ulcer treatment in TCM is affected by factors such as trends, cycles, and mutations, which are complex and changeable, prediction research on medication for peptic ulcer treatment in TCM needs to be conducted based on full data mining information. Therefore, data mining and prediction research based on time series decomposition of peptic ulcer medication are carried out to provide technical support for decision making in the management of peptic ulcer medication resources.

RETRACTED

In this study, a neural network model which is based on time series decomposition is developed to ensure mining and prediction medication pattern of peptic ulcer treatment in Chinese medicine. The cumulative distance level method, Mann–Kendall trend analysis method, Hurst exponent method, and characteristic point method are used for trend analysis. The wavelet analysis method was used for periodicity analysis and Mann–Kendall mutation test and Pettitt methods are used for mutability analysis. Autocorrelation and unit root methods are used to test the random terms. The Chinese herbal formulas (where the main diseases are peptic ulcer, peptic ulcer, cerebral leakage, and cerebral abscess) are collected from the databases of medicine wisdom and modern application of prescriptions. Furthermore, methods of frequency analysis, association rule analysis, and factor analysis are used to evaluate the grouping pattern of prescriptions for peptic ulcer treatment. The error in the proposed scheme between the predicted and the measured values of 87 prescriptions, which involve five Chinese medicines for peptic ulcer and 160 Chinese medicines, obtained from the neural network was 16.79%.

The remaining paper is organized described as follows: In the subsequent section, data processing methodology is presented which depicts how the collected data is processed. In Section 3, the proposed methodology is presented in detail which is followed by the results section where performances of the proposed and the existing state-of-the-art methods are compared. In Section 5, generalized discussion on the possible usage of the proposed methodology with respect to the existing methods is presented. Lastly, concluding remarks are given.

## 2. Data Processing

With the pivot table function of Microsoft Office Excel 2017, we have statistically analyzed the frequency, efficacy, and aptitude of the Chinese medicines using CytoNCA [5] and plug-in Cytoscape 3.7.2. We have filtered the core Chinese medicines based on the attribute values of degree centrality (DC), betweenness centrality (BC), and closeness centrality (CC). The important nodes that were greater than two times the median of node DC are screened for the first time. Every attribute value is greater than their respective medians in the second screening. The Apriori algorithm of IBM SPSS Modeler 18.0 is used to set the conditions of support ≥20%, confidence ≥60%, and the maximum number of previous terms of 5, etc., to mine the potential association rules among TCMs and visualize them. IBM SPSS Statistics 25.0 is used to conduct factor analysis of TCMs and the maximum variance method is selected for factor analysis to obtain eigenvalues >1. The maximum variance method was chosen to obtain the common factors with eigenvalues >1.

RETRACTED

## 3. The Proposed Mechanism

In this paper, we have developed a neural network model which is based on the time series decomposition to ensure mining and prediction medication pattern of peptic ulcer treatment in Chinese medicine. Various sections of the proposed methodology are presented below.

### 3.1. Time Series Method

The medication used in the treatment of peptic ulcer in Chinese medicine is influenced by various factors and has various variation characteristics such as trend, periodicity, and mutation. Decomposing the time series into trend, periodicity, mutation, and random terms and analyzing these terms can better reveal the variation pattern of medication data of peptic ulcer. Let *X* be a time series, *T* be a trend term, P be a periodic term, B be a mutation term, and *R* be a random term; then, *X* can be expressed as

(1) $$\begin{array}{c} X=T+P+B+R. \end{array}$$

- Common trend term analysis methods include cumulative distance level [6], Mann–Kendall trend analysis [7], Hurst exponent [8], and Eigen point [9]
- Period term analysis methods include wavelet analysis [1]
- Mutation term analysis methods include Mann–Kendall mutation test [10] and Pettitt mutation test
- Random term test methods include autocorrelation plot and unit root.

### 3.2. A Time Series Decomposition-Based Data Mining Prediction Model for Peptic Ulcer Medication Use

A data mining and forecasting model (DMAF) which is based on time series decomposition is proposed. This model can not only mine the intrinsic information of TCM medications for peptic ulcer treatment but also make accurate prediction:

- Data mining (data decomposition): for the Chinese medicine treatment of peptic ulcer medication *X*, the trend term *T* is decomposed by the characteristic point method. The periodic term P is decomposed by the wavelet analysis method. The Mann–Kendall and Pettitt methods are used for mutability analysis, and the mutation term B is not considered without special circumstances. The residual term X-T-P-B is calculated to obtain the random term *R*.
- Data mining (cumulative method): the Mann–Kendall trend analysis method, the Hurst index method, and the characteristic point method are used for trend analysis. The wavelet analysis method is used for periodic analysis whereas Mann-Kendall and Pettitt method are used for mutation analysis and random term *R* is calculated.
- Data mining (trend analysis): it is performed by the cumulative level method, Mann-Kendall trend analysis method, Hurst index method, and characteristic point method. Period analysis is performed by the wavelet analysis method, mutability analysis is performed by the Mann-Kendall and Pettitt methods, and the random term was tested by the autocorrelation graph and unit root methods, respectively.
- Data prediction: for data prediction, the linear extension method is used to extend the trend term *T* based on the end line of the characteristic point method to obtain *T*_*y*_ and the Matlab wavelet toolbox extend function is used to extend the period term P to obtain *P*_*y*_. Then, the extended trend term *T*_*y*_ , the periodic term *P*_*y*_, and the predicted random term *P*_*y*_ are added together to obtain the prediction results, as shown in Figure 1. To improve the prediction accuracy, the NAR neural network is optimized by genetic algorithm and the flowchart is shown in Figure 2.

RETRACTED

## 4. Experimental Results and Evaluations

In this section, a detailed and comparative analysis of the proposed and existing state-of-the-art approaches is presented in terms of various results obtained through the experimental process.

### 4.1. Classification

In the modern application database of prescriptions, 62 and 20 prescriptions were retrieved with the keyword “peptic ulcer,” respectively. Five (5), thirty (30), and six (6) prescriptions were retrieved with the keyword “peptic ulcer” in the database of medicine wisdom, respectively. The remaining keywords were not retrieved. After screening and deduplication, 87 prescriptions meeting the criteria were obtained. According to the efficacy of the formulas and the “Chinese Medicine Clinical Terminology—Evidence Section,” the disease types involved in the formulas were determined, among which the most formulas corresponded to wind-heat in the lung meridian (39 times) and damp-heat in the spleen and stomach (19 times), as shown in Figure 3.

### 4.2. Frequency, Taste, and Attribution

The eighty-seven (87) study prescriptions have involved 160 herbal medicines and were used 800 times. The efficacy of these herbal medicines is that they are mostly heat-clearing and deficiency-supplementing medicines, which are shown in Table 1. The distribution of their sexual tastes and meridians is shown in Figure 4.

RETRACTED

### 4.3. Core Chinese Medicine Screening

Seventeen (17) core herbs are shown in Table 2 with their specific frequency of use and efficacy. The most frequently used herbs were Bai Zhi (48 times), Xin Yi (48 times), and Cang Er Zi (39 times), which were used as antiphlogistic herbs, Licorice (45 times) as deficiency tonic, and *Scutellaria* (39 times) as heat-clearing herbs.

### 4.4. Analysis of Association Rules

It is evident from Figure 5 that the classification of peptic ulcer types includes the most frequent cases of wind-heat in the lung meridian and damp-heat in the spleen and stomach. Therefore, these two types of evidence are used as representatives for in-depth analysis of the pattern of medication in the treatment of peptic ulcer with Chinese medicine.

The IBM SPSS Modeler 18.0 software was used to analyze the association rules for the prescriptions involved in the 2 evidence types, based on the support degree of the commonly used high-frequency herbal combinations. The association rules of herbal medicines are shown in Figures 6 and 5, respectively, where size of nodes represents the degree. Thickness of connecting lines indicates the degree of association. We have observed that, in treatment of pulmonary meridian wind-heat type peptic ulcer, node degree values among the herbs Xin Yi, Bai Zhi, and Cang Er Zi are the highest. Herbal combinations composed of these have the strongest degree of association. Similarly, *Glycyrrhiza glabra*, Xin Yi, Bai Zhi, and Chuan Xiong are key combinations for peptic ulcers of the damp-heat type of the spleen and stomach.

### 4.5. Factor Analysis

KMO and Bartlet's spherical test have showed that both lung meridian wind-heat type and spleen-stomach damp-heat type data were suitable for factor analysis. Using principal component analysis (PCA), the results showed that six common factors were extracted for both types of data. The cumulative factor contribution of the lung meridian wind-heat type data was 68.10%, and the cumulative factor contribution of the spleen-stomach damp-heat type data was 83.04%. This indicates that the extracted common factors could reflect all the information involving traditional Chinese medicines. Each Chinese medicine was grouped into the common factor with the highest contribution value [6]. Its rotated component matrix loadings are shown in Figures 7 and 8.

## 5. Discussion and Evaluation

Su Wen has proposed that the pathogenesis of peptic ulcer is wind-heat in the lung meridian. Sui Dynasty Chao Yuan Fang's “Treatise on the Origin of Diseases” believed that the occurrence of peptic ulcer is due to “qi deficiency by wind and cold in the mind.” Zhang Jingyue believed that overeating fatty, sweet, greasy, and hot food causes spleen and stomach peptic ulcers. The peptic ulcer is caused by the heat of the spleen and stomach caused by excessive consumption of fatty, sweet, greasy, and hot foods. In modern Chinese medicine, it is believed that peptic ulcers are invaded by wind-cold or wind-heat evil, resulting in loss of lung circulation and loss of nasal orifices. If the evil is not resolved, it is damp-heat into the lungs for a long time, resulting in abnormal spleen and stomach transportation, clear yang does not rise, cloudy yin does not descend, and dampness is heavy and sticky, causing repeated attacks and stagnation. Peptic ulcer is an evidence of deficiency and standard reality, and the actual evidence includes wind-heat in the lung, heat in the biliary organs, and damp-heat in the spleen and stomach. Deficiency evidence includes deficiency cold in the lung and weakness in the spleen. The treatment should be external removal of superficial evil, elimination of blood stasis and elimination of turbidity, internal regulation of the internal organs, and clearing heat and dampness [7].

RETRACTED

It was observed that 87 prescriptions involved a total of five peptic ulcer evidence types among which the lung meridian wind-heat type and spleen and stomach damp-heat type corresponded to most of the treatment prescriptions. The results of the analysis of the frequency and nature of the Chinese medicines showed that 160 Chinese medicines were used 800 times in total among which the most frequent use was for relieving symptoms, clearing heat, and notifying deficiency. Rong et al. [8] analyzed the TCM evidence types and elements of symptoms of peptic ulcer and found that, in the early stage of peptic ulcer, the superficial evil such as heat, dampness, wind, and cold invaded the nasal orifices and the actual evidence was predominant, while in the later stage of the disease, the deficiency and reality were mixed. Therefore, the application of antiphlogistic drugs, heat-clearing drugs, and deficiency-supplementing drugs in the treatment of peptic ulcer is assumed to be in accordance with the drug evidence. The analysis of the nature and taste of the meridians shows that most Chinese medicines are cold, warm, pungent, and bitter to the lung meridians or warm and pungent to the spleen meridians. “Identification” records that “peptic ulcer has two original symptoms of cold and heat, which are not only caused by Gallbladder Heat. Heat is solid heat and cold is deficiency cold. Cold medicine should be used for heat and mild agent for cold.” However, “Materia Medica” includes “bitter, diarrhea, dryness, firmness, pungent, powder, moistening and moving.” It also believes that bitter traditional Chinese medicine has the characteristics of purging heat, drying dampness and strengthening Yin, and is mostly used to treat heat, fire, and dampness syndrome. Pungent Chinese medicine has the effect of dispersing and relieving the surface, moving qi and blood. The theory of “the lung is open to the nose” in Chinese medicine indicates that the treatment of nasal diseases should first be started on the lung. Chen Leping and others [9] also found that peptic ulcer disease includes multiple internal organs such as lung, spleen, stomach, and gallbladder. Thus, herbs with cold and warm properties and pungent and bitter taste and belonging to the lung and spleen meridians are able to address the cause of the disease and directly attack the disease.

RETRACTED

It is evident that, in the clinical treatment of peptic ulcer, we should pay attention not only to the prescription of drugs, but also to the identification of evidence and rational use of drugs to achieve the effect of both primary and secondary treatment. In summary, this study systematically analyzed the peptic ulcer typology and the medication rules of its therapeutic prescriptions. Furthermore, it clarified the dispensing characteristics and formulas rules of peptic ulcer therapeutic prescriptions. It has provided medication ideas and references for the clinical treatment of peptic ulcer.

## 6. Conclusions

In this paper, a neural network model which is based on time series decomposition was developed to enable mining and accurate prediction of the medication pattern of peptic ulcer treatment in Chinese medicine. The autocorrelation and unit root methods were used to test the random terms. The Chinese medicine prescriptions whose main diseases were peptic ulcer, peptic ulcer, cerebral leakage, and cerebral abscess were collected from the database of medicine wisdom and modern application of prescriptions. Methods of frequency analysis, association rule analysis, and factor analysis were applied to explore the grouping pattern of prescriptions for the treatment of peptic ulcer. In this paper, the error between the predicted and the measured values of 87 prescriptions, involving five Chinese medicines for peptic ulcer and 160 Chinese medicines, obtained from the neural network was 16.79%.

In future, we will try to enhance the proposed neural network-based model for other diseases and medication procedures.

## Figures and Tables

**Figure 1:** Flowchart of the study.

**Figure 2:** Flowchart of neural network optimization based on genetic algorithm.

**Figure 3:** Distribution of evidence of peptic ulcer.

**Figure 4:** Heat map of Chinese herbal medicine for peptic ulcer treatment.

RETRACTED

**Figure 5:** Association rules for the lung meridian and wind-heat type.

**Figure 6:** Association rule of damp-heat type of the spleen and stomach.

**Figure 7:** Lung meridian wind-heat type load diagram.

**Figure 8:** Load diagram of the spleen and stomach damp-heat type.

**Table 1:** Classification of frequency and efficacy of Chinese herbal medicines for peptic ulcer treatment.

No.	Effect	Frequency
1	Solution table	280
2	Clearing heat	170
3	Tonifying deficiency	140
4	Resolving phlegm, relieving cough, and relieving asthma	53
5	Promoting blood circulation and removing blood stasis	42
6	Diuresis and dampness	30
7	Dehumidification	17
8	Astringency	12
9	Dispelling wind dampness	12
10	Calming liver and calming wind	12
11	Regulating qi	11
12	Enlighten	11
13	Wenli	3
14	Hemostasis	3
15	Purgation	2
16	Attacking poison, killing insects, and relieving itching	2

**Table 2:** Frequency and efficacy of core herbs.

	Traditional Chinese medicine	Frequency	Effect
1	*Angelica dahurica*	48	Solution table
2	*Magnolia*	48	Solution table
3	Licorice	45	Tonifying deficiency
4	*Xanthium sibiricum*	39	Solution table
5	Baikal skullcap	39	Clearing heat
6	Rhizome of chuanxiong	28	Huoxue huacha
7	Mint	24	Solution table
8	Chinese bellflower	24	Resolving phlegm, relieving cough, and relieving asthma
9	*Asarum*	21	Solution table
10	Windbreak	18	Solution table

## Data Availability

The datasets used and analyzed during the current study are available from the corresponding author upon reasonable request.
